The article "On the networking synthesis of studio factors to the integration of design pedagogy" was retracted in 2025. Reasons: unreliable results or conclusions; concerns about the peer review; concerns about the article.

# On the networking synthesis of studio factors to the integration of design pedagogy

**DOI:** 10.1371/journal.pone.0212177

**Published:** 2019-03-06

**Authors:** Zheng-Hui Wang, Xin Li, Shih-Chih Chen, Chiu-Shui Chan, Penny Lewis, Ihab Hijazi

**Affiliations:** 1 School of Urban Design, Wuhan University, Wuhan, China; 2 Department of Information Management, National Kaohsiung University of Science and Technology, Kaohsiung City, Taiwan; 3 College of Design, Iowa State University, Ames, IA, United States of America; 4 Department of Architecture and Urban Planning, University of Dundee, Dundee, United Kingdom; 5 Urban Planning Engineering Department, An-Najah National University, Nablus, Palestine; University College London, UNITED KINGDOM

## Abstract

Studio is critically important for design education, but few attempts have been made to demonstrate the parallels between studio factors and design performance. This paper adopts a coherent set of analyses to investigate the major studio factors and attempts to quantify the networking interactions among them. First, it describes how architectural studio is usually organised based on some major factors. Next, a theoretical model is established according to the described hypotheses and their mutual interactions. Third, the research method and statistical analysis with structural equation modelling (SEM) are presented. Finally, the results of this empirical examination are presented for discussion and suggestions. Our findings reveal that studio tutorials have no significant effect on undergraduate's design performance. In contrast, students’ subjective intention plays a more important role in shaping their behaviour, indicating the importance of transferring those exterior forces into internal benefits when the studio instructor attempts to optimise the pedagogy. These findings are also inspiring for all creative disciplines.

## 1. Introduction

Architectural design involves a series of space-based problem-solving activities requiring decision making processes to meet human needs [1]. It involves cognitive abilities such as intuition, imagination, and creativity [2]. Unlike other disciplines that have been taught in the current university system, the architecture curriculum is organised around studio and project work. Studio has long been a part of architectural education and it provides a framework for many other creative disciplines [3]. Students of creative disciplines such as architectural design, industrial design and fine arts usually spend most of their time working, studying, and even living in the design studio where they have highly intensive interactions with tutors and other students [4, 5]. Improving the pedagogy of design studios is critical for all creative disciplines and could help students to acquire more of the professional skills needed to become efficient designers and independent citizens [3, 6].

The article "On the networking synthesis of studio factors to the integration of design pedagogy" was retracted in 2025. Reasons: unreliable results or conclusions; concerns about the peer review; concerns about the article.

Design education aims to facilitate the effective acquisition of design expertise for undergraduates. It extends their professional acumen, technical knowledge, critical thinking, civic responsibility and social cognition. Although research on professional teaching has been a major focus of creative disciplines in higher education [7, 8, 9], qualitative studies on design studios and their corresponding influence on students’ learning behaviours are insufficient. Ji (2017) attempted to employ some possible factors that influence how students learn to design, such as creativity, spatial ability and visual cognitive style; however, the result has shown insignificant correlations [10]. Some scholars argue that design that follows a step-by-step process of prescribed methodology does not necessarily guarantee a successful result [11]. Design activities are difficult to define because of the complicated process involving student predisposition and motivation, the quality and expertise of design instructors, the teaching method and instruction strategy. In studio, the learning process of design studio is determined by various factors, such as descriptions and conditions for a specific project (the design brief), design-based explorative research around a given topic (design research), education background of instructors (instructor quality), the quality and effectiveness of their instruction (studio tutorial), and their comments on a design work for optimisation (review feedback). These issues have been discussed in previous studies around similar topics, such as studio teaching and curriculum [12], design critiquing and reviewing [13], instructor-student relationships [14], and other general issues [15, 16, 17]. However, these previous studies might have neglected to create a systematic framework for exploring the relationships among these critical factors and their influences on students' motivation of participating in design study. To the best of our knowledge, how these factors influence each other is unknown, as is the corresponding comprehensive synthesis that influences students' involvement in design work.

In order to fill these knowledge gaps, this research aims to address the process and relevant mechanisms that influence students' design performance with the remainder of this paper. Section 2 describes the organisation and composition of the design studio, then a theoretical model indicating various hypotheses and corresponding variables is established. In Section 3 and 4, the method and analysis process are presented. From Section 5 to 7, the results of the empirical examination are presented, followed by a discussion, implications and coping suggestions.

The article "On the networking synthesis of studio factors to the integration of design pedagogy" was retracted in 2025. Reasons: unreliable results or conclusions; concerns about the peer review; concerns about the article.

## 2. Literature review

### 2.1 Design studio

The studio is a place where design instructions are instilled in students for developing creative ideas and design concepts. In the studio, students gain theoretical knowledge and a practical basis to forge judgements about their design products [5]. To a large extent, the modern design studio is structured based on a traditional French prototype of Ecole des Beaux Arts atelier, which emphasises the training of classical experience and knowledge [18, 19]. In the twentieth Century, the Bauhaus’s ethos of ‘learning by doing’ and interdisciplinarity made an impact on studio culture and more recently an element of apprenticeship has been introduced to shape the modern structure of architectural design studio.

### 2.2 Motivation and design performance

In most university subjects, academic performance is usually measured by the grading of courses and tests. Science-based courses such as math or physics, measure the objective accuracy of a student’s work, but architectural design involves the subjective assessment of both the students’ development work and their final submission. In architecture studio, the assessment appraises design concepts, design development, and graphic presentation according to the course focus and objectives [20]. This approach is not without its critics; within architecture departments there is an ongoing debate about whether students with higher grades will eventually become successful professional designers in the future [21]. Actually, performance in design studies is based on various factors, such as student motivation, teacher impact, and the school’s particular interests [22]. Among these factors, motivation is the most valuable characteristics that spur and drive one's behaviour by converting the exterior forces into the internal objective. Motivation plays a critical role in shaping one's design performance and is important for any instructional design [23]. Accordingly, the professor in educational psychology Keller [24, 25] has studied learner motivation in undergraduate courses and developed the ARCS model which looks at motivation in terms of four factors: attention, relevance, confidence, and satisfaction [26].

**Hypothesis 1:** Design Motivation (DM) has a positive effect on undergraduates' design performance (GR).

### 2.3 Design brief

For a design project, teachers often start with lectures or presentations describing the proposed project. The project ‘brief’ outlines a specific problem to be solved or specific issues that demand an innovative design solution, in much the same way as a planning brief would be produced in the professional world. The attributes of the project such as location, context, surrounding conditions, and user's profile determine the level of complexity of the project and the difficulty that it poses to designers [27]. Unlike scientific courses in which problems are often precisely defined so that students can take a series of steps in a process to arrive at the singular solution, design cannot be solved using only calculations based on formulas and there may exist alternative satisfactory solutions, even though some technical aspects of a design problem may be predictable within certain limits. The design project usually poses an open range of demands and multivariable problems. Designers and clients have to clarify different needs without knowing precise answers, whereas the solutions are often expected to be original and creative [28]. Design projects encourage students to develop critical thinking and questioning until they reach proper solutions, both “found” and “created” [28]. Through the course of a student’s design education, the problems presented in studio gradually become more complex and open-ended as more factors are included for consideration. The aim of the studio project is not merely for providing solutions, but also for cultivating curiosity and interest that help students develop personalized design methodologies.

The article "On the networking synthesis of studio factors to the integration of design pedagogy" was retracted in 2025. Reasons: unreliable results or conclusions; concerns about the peer review; concerns about the article.

**Hypothesis 2:** The Design Brief (DB) has a positive effect on Design Motivation (DM).

**Hypothesis 3:** The Design Brief (DB) has a positive effect on Studio Tutorial (ST).

### 2.4 Design research

The trend towards research-led education has gained increasing attention in the modern design pedagogy. Reports on student's learning difficulties often highlight the lack of a comprehensive understanding of the problem and the corresponding research process to eliminate confusion [29]. This implies an implicit need among students to undertake research methodologies [30]. Therefore, instructional approaches combining project assignment and allowing undergraduates to engage in the design research process would be helpful to broaden students’ interests, maintain positive study attitudes, increase their dedication to intensive study, and promote ability of creative and reasonable decision making [31].

**Hypothesis 4:** Design Research (DR) has a positive effect on Design Motivation (DM).

### 2.5 Studio tutorial and instructor quality

The traditional design studio purposely adopts a trial-and-error approach based on the philosophy of practice-in-reflection [32]. According to this method, design work is carried forward by means of mock-ups, drawings, sketches, and digital images. In different sessions, students reflect on their design ideas to play with different materials and tectonic composition until they find the most satisfying proposal from many alternatives [32]. The ongoing process is supervised by qualified instructors once or twice a week. Instructors are responsible to guide students for better solutions and keep the studio in good order [33, 34]. Instructors might consider various forms of teaching, including desk talk, case study, lecture, presentation, and demonstrations. Suggestions are offered for proper modifications based on careful assessment of students' design trials [35, 36]. Sometimes the instructor acts as a master to impart professional knowledge and experience. And other times, the instructor also adopts a user-designer relationship to give comments and demands from a user's perspective [37]. The teacher is often the studio organiser who facilitates collaborative learning among students. All three models rely heavily on the teachers' merits, such as educational background, academic capability, experience, and communication skills. Therefore, both the perceived quality of the instructor from students' perspective and perceived teaching quality should be considered as important determinants that influence students' design behaviours. Therefore, the instructor quality refers to the perceived quality of the instructor from students' perspective, and studio tutorial refers to the evaluation to the effectiveness of teaching.

The article "On the networking synthesis of studio factors to the integration of design pedagogy" was retracted in 2025. Reasons: unreliable results or conclusions; concerns about the peer review; concerns about the article.

**Hypothesis 5:** Studio Tutorial (ST) has a positive effect on Design Motivation (DM).

**Hypothesis 6:** Studio Tutorial (ST) has a positive effect on Design Performance (GR).

**Hypothesis 7:** Instructor Quality (IQ) has a positive effect on Studio Tutorial (ST).

### 2.6 Review feedback

Besides regular studio tutorial from teachers, reviews and ‘public’ critiques are the major forces that help students to move their studies forward [38]. The open review critique or ‘crit’ can take various forms including desk crits, pin-ups, juries, and reviews [39]. During different sessions of the regular class, students may have to present their work to teachers and occasionally to guests for critiques to receive suggestions for further development. Students are encouraged to attend the crits and reviews of their peers as they will learn by being exposed to a general discussion of design problems and solutions. They may become more confident regarding their work, and sometimes frustrated if they encounter negative comments. Both results will influence a student’s next move.

The article "On the networking synthesis of studio factors to the integration of design pedagogy" was retracted in 2025. Reasons: unreliable results or conclusions; concerns about the peer review; concerns about the article.

**Hypothesis 8:** Review feedback (RF) has a positive effect on design intention (INT).

**Hypothesis 9:** Review feedback (RF) has a positive effect on studio tutorial (ST).

### 2.7 Structuring the theoretical model

Our theory is established according to the above hypotheses based on an analysis of the framework of studio organisation and evidence from literature review. A construct is the conceptual term which is used to constitute a theory and also serves as a surrogate to describe a real phenomenon [40]. In this study we have identified six constructs describing the major factors affecting studio teaching and learning. They are defined as: Design Brief (DB), Design Research (DR), Review Feedback (RF), Instructor Quality (IQ), Studio Tutorial (ST), and Design Motivation (DM). Design performance (GR) is listed as an independent variable. Finally, a theoretical model containing all these constructs is established to test the complexity and interactions among the described factors in studio, the networking synthesis on students' intention of participation in design work, as well as the influence on design performance (Fig 1).

**Fig 1:** Theoretical research model.

## 3. Methodology and data

### 3.1 Instrument

This research used a multi-item measurement for each construct via the following steps. First, all the constructs and the corresponding measure items were defined based on the framework of studio organisation and literature evidence to adapt the research context. Second, items were measured by questionnaires. After the questionnaire was drafted, a pre-test was performed to eliminate certain terminology and ambiguous expressions, ensuring the questions could be easily understood by formal participants. Finally, twenty-seven items for measuring the six constructs except GR were selected. For all items, a seven-point Likert scale measurement was used ranging from strongly disagree (1) to strongly agree (7). We measured GR with converted seven-point Likert scale from the hundred percentage point score of the respondent (60–65 = 1; 65–70 = 2; 70–75 = 3; 75–80 = 4; 80–85 = 5; 85–90 = 6; above90 = 7; no respondent reported the score under 60).

### 3.2 Data collection

The random sampling was conducted to collect data via an online survey that lasted for three weeks. A total of 241 undergraduate students in a five-year architecture programme were involved in this research. The students were from fifteen major universities in China, ranked at all levels according to national programme accreditation results in 2016. Each respondent received a lottery ticket offering the opportunity to get a coupon as a token of gratitude. There is no potential harmful indication to subject's biological identification and one's interests in our study. All subjects have been properly instructed and privacy and anonymity of the collected data is guaranteed. The written consents have been obtained from all the participants according to the principles of Declaration of Helsinki. The process has been reported to the IRB of school of urban design at Wuhan University, and an approval has been issued. The sample demographics are listed in Table 1. From the raw data, 11 participants were removed due to errors found in the data, and eventually 230 participants were selected for the final report, resulting in 100 males (43.5%) and 130 females (56.5%). Among the selected respondents, 26 were first-year students (11.3%), 57 were second-year students (24.8%), 84 were third-year students (36.5%), 45 were fourth-year students (19.6%), and 18 were fifth-year students (7.8%). All the data comply with the statistical requirements.

The article "On the networking synthesis of studio factors to the integration of design pedagogy" was retracted in 2025. Reasons: unreliable results or conclusions; concerns about the peer review; concerns about the article.

**Table 1:** Demographic attributes of the respondents.

	Category	Number	Percentage
Grade	1st Year	26	11.3
	2nd Year	57	24.8
	3rd Year	84	36.5
	4th Year	45	19.6
	5th Year	18	7.8
Gender	Male	100	43.5
	Female	130	56.5

Data entry was checked to ensure the absence of outliers or missing values for the measure item variables. The approximate normality was examined beforehand: no non-normality was found when items were examined for skewness and kurtosis, whose absolute value should meet the criteria of < 3 and <7, respectively [41] (Table 2). A coherent logical analytical process is as follows: confirmatory factor analysis (CFA), testing of composite reliability, testing of convergent validity and discriminant validity, model testing and modification, interpretation and discussion of the model estimates.

**Table 2:** Normal distribution test for the constructs.

	GR	DB	DR	RF	IQ	ST	DM
Mean	5.34	4.40	5.39	4.53	4.59	5.04	5.20
Std. Deviation	1.19	1.20	1.12	1.31	1.38	1.18	1.41
Skewness	-1.17	-.58	-1.23	-.81	-.47	-1.06	-1.22
Kurtosis	1.97	.01	1.83	.00	-.25	.82	1.29

### 3.3 Structural equation modelling

Structural equation modelling (SEM) was used to test the relationships among examined constructs and provide evidence to improve the proposed theory [42, 43]. SEM adopts the variance-covariance matrix with raw data when loading the input [44] and enables the modelling of constructs while taking the loading of measured items into account to enhance calculation reliability by avoiding inaccurate standard errors [45]; these errors have no influence on the overall goodness-of-fit indices (GFIs) and parameter estimates of the model [44].

Confirmatory factor analysis (CFA) was employed for all the latent variables within each construct. The reliability and validity should meet the required criteria before conducting a structural model for regression analysis. Then, a structural model was established. If the model fit was accepted, multiple regressions were applied for path analysis to estimate the alignment between designated constructs.

The article "On the networking synthesis of studio factors to the integration of design pedagogy" was retracted in 2025. Reasons: unreliable results or conclusions; concerns about the peer review; concerns about the article.

## 4. Analysis process

### 4.1 Confirmatory factor analysis

Confirmatory factor analysis (CFA) was conducted following the procedure set forth by Gerbing & Hamilton [46], extracting the common variance into a single factor. According to Hair's recommendation [47], the item loadings (*λ)* of each construct should be at least 0.5, and the cut-off factor loading is 0.60, while items with cross-loadings over 0.4 should be rejected as a means of item juxtaposition among several constructs. Meanwhile, the value of Kaiser-Meyer-Olkin (KMO) is calculated to meet the requirement of being close to 0.6 or higher [41]. After examination, all standardised item loadings of the constructs are listed (Table 2), and the KMO of all constructs are also mostly higher than 0.7, meeting both requirements for further analysis.

### 4.2 Composite reliability

The internal consistency of all items within each construct was measured using the measure of composite reliability (Cronbach's α), whose value should be within the domain of 0.7 and 0.9, and the value of corrected item-total correlation should be at least 0.5 as suggested by Nunnally & Bernstein [48]. For composite reliability, a value above 0.9 might indicate a collinearity among several items that necessitates careful review from other indices to determine a cut-off. During the examination, inappropriate items are discarded from all constructs except IQ according to the described standard. The Cronbach's α for DM is justified for maintenance at 0.92 because cutting more items will result in low KMO and unexpected loss of information. At that point, the calculation is repeated until composite reliability is within a proper domain (Table 3), indicating an acceptable internal consistency for the next step analysis.

**Table 3:** Result of the confirmatory factor analysis and composite reliability.

Construct Items		Factor Load	Construct Correlation Matrix Items						Statistical Test		
									Item-Total	Cronbach's α	KMO
DP			DP1	DP2	DP3	DP4			l		
	DP1	0.83	1						0.66	0.80	0.70
	DP2	0.85	0.65	1					0.7		
	DP3	0.80	0.52	0.55	1				0.63		
	DP4	0.76	0.47	0.51	0.5	1			0.58		
RD			RD1	RD2	RD3	RD4					
	RD1	0.84	1						0.69	0.85	0.72
	RD2	0.68	0.39	1					0.49		
	RD3	0.88	0.72	0.45	1				0.76		
	RD4	0.85	0.6	0.47	0.67	1			0.71		
RF			RF1	RF2	RF3	RF4	RF5	RF6			
	RF1	0.76	1						0.63	0.87	0.82
	RF2	0.81	0.64	1					0.71		
	RF3	0.78	0.44	0.61	1				0.67		
	RF4	0.84	0.6	0.56	0.54	1			0.74		
	RF5	0.83	0.56	0.57	0.50	0.74	1		0.73		
	RF6	0.60	0.22	0.35	0.56	0.38	0.42	1	0.47		
IQ			IQ1	IQ2	IQ3	IQ4					
	IQ1	0.84	1						0.72	0.88	0.73
	IQ2	0.90	0.7	1					0.81		
	IQ3	0.90	0.63	0.72	1				0.81		
	IQ4	0.93	0.67	0.78	0.86	1			0.87		
ST			ST1	ST2	ST3	ST4					
	ST1	0.84	1						0.74	0.90	0.84
	ST2	0.90	0.71	1					0.83		
	ST3	0.90	0.66	0.79	1				0.80		
	ST4	0.93	0.62	0.69	0.68	1			0.74		
INT			INT1	INT2	INT3	INT4					
	INT1	0.85	1						0.79	0.92	0.76
	INT2	0.91	0.81	1					0.80		
	INT3	0.90	0.77	0.79	1				0.77		
	INT4	0.85	0.31	0.31	0.29	1			0.33		

The article "On the networking synthesis of studio factors to the integration of design pedagogy" was retracted in 2025. Reasons: unreliable results or conclusions; concerns about the peer review; concerns about the article.

### 4.3 Data Validation

Convergent validity testing was applied to examine whether all items share significant commons on the same construct. The convergent validity would also reconfirm the qualification of confirmatory factor analysis. Three criteria should be met simultaneously as Fornell & Larcker suggest [49]: (1) all the item loadings are significant and exceed 0.7; (2) the composite reliabilities exceed 0.80, and (3) the average variance extracted (AVE) by each construct exceeds 0.50. According to results presented in Table 3, the *λ*-values of all twenty-seven items of the six constructs were between 0.75 and 0.94 and significant at p<0.001, exceeding the minimum requirement. The Cronbach's α values of all six constructs were within 0.8 for the construct of RD and 0.92 for the construct of INT. The AVE values for all constructs ranged between 0.72 for design project and 0.86 for design intention, well above the minimum threshold of 0.50, indicating the assured convergent validity for all constructs.

The discriminant validity testing was applied to examine whether individual items could be adequately distinguished from different constructs. The standard requires that the square root of AVE of each construct be higher than the correlation with other constructs in the CFA model [49]. Values in bold along the principal diagonal in Table 4 indicate that the square root of the AVE of each construct was higher than the corresponding correlations of other constructs, namely, the off-diagonal elements in the corresponding rows and columns, assuring discriminant validity since this construct is more closely related to its measured items than with the other constructs.

**Table 4:** Results of the validity test.

Construct	Convergence Validity	Discriminate Validity						Descriptive Statistics		
	AVE	DP	RD	IQ	RF	ST	INT	Mean	Std. Deviation	N
DP	.72	**.85**						4.40	1.20	230
RD	.78	.29	**.88**					5.39	1.12	230
RF	.66	.61	.32	**.81**				4.53	1.31	230
IQ	.81	.49	.05	.63	**.90**			4.59	1.38	230
DI	.77	.61	.23	.70	.69	**.88**		5.04	1.18	230
INT	.86	.52	.43	.49	.34	.54	**.93**	5.20	1.41	230

The items on the diagonal represent the square roots of the AVE; off-diagonal elements are the correlation estimates

The article "On the networking synthesis of studio factors to the integration of design pedagogy" was retracted in 2025. Reasons: unreliable results or conclusions; concerns about the peer review; concerns about the article.

## 5. Results

### 5.1 Model-fit estimation

The proposed structural model was tested with AMOS 22 using the maximum likelihood estimation. First, the coefficients of determination (*R*^*2*^*)* were estimated for all items representing the percentage of explained variance within each construct. The goodness-of-fit indices were calculated for the structural model, as the same GFIs would be applied in assessing the measurement model. Second, the hypothesis of each path was estimated with the standardised path coefficients and their statistical significance. Finally, the coefficient of determination (*R*^*2*^*)* was also applied for each construct or independent variable to the percentage of explained variance. Instead of evaluating each index independently in multiple regression analysis, a variety of goodness-of-fit indices were combined to meet the model-fit criteria, which determines the degree to which the sample variance-covariance data fit the structural equation model. For instance, some major requirements are as follows: (1) Ratio of chi-square to degree of freedom (χ^2^/df) <3; (2) GFI > 0.90 and AGFI > 0.80 (acceptable) or 0.90 (good) and; (3) either CFI > 0.90 or RMSEA < 0.06 [50]. Table 5 presents other model-fit estimates as well as the recommended criteria. Except for AGFI, all the model-fit estimates exceeded the recommended level of acceptance. MacCallum & Hong [51] argue that AGFI could be acceptable at a 0.80 level because of its inherent sensitivity to a large sample size. Correlations might exist between the estimate errors and other constructs ort variables, resulting in a high chi-square value which compromises the model-fit.

**Table 5:** Model-fit criteria and the test results.

Model-fit	χ^2^/df	GFI	AGFI	RMSEA	CFI	NFI	RFI	IFI	TLI
Standard	<3	>0.9	>0.8	<0.08	>0.9	>0.9	>0.9	>0.9	>0.9
Initial	2.17	0.82	0.78	0.07	0.91	0.85	0.83	0.91	0.90
Modified	**1.53**	**0.91**	**0.88**	**0.05**	**0.97**	**0.92**	**0.91**	**0.97**	**0.97**

Note: root mean square error of approximation (RMSEA); goodness-of-fit index (GFI); adjusted goodness fit index (GFI); comparative fit index (CFI); normed fit index (NFI); relative fit index (RFI); incremental fit index (IFI); Tucker-Lewis index (TLI)

The model-fit was close to the requirement for the initial model which contained all twenty-seven items (Table 5) except some model-fit indices. To increase the goodness-of-fit indices, the chi-square value should be reduced by cutting two redundant errors and the corresponding measuring items. As a result, a set of goodness-of-fit indices in Table 5 satisfies the combination rule as well as the independent level of recommended fits. Thus, the result indicates that the proposed model has a good model-fit with GFIs being all within the acceptable standards, χ^2^/df (672.80/310 = 2.17), GFI (0.82), AGFI (0.78), NFI (0.85), CFI (0.91), and RMSE (0.07). Through model modification of cutting two items from RF, the AGFI is increased to 0.88, which qualifies as an acceptable level and brings it close to an ideal situation. The following values indicate an improvement of goodness-of-fit indices both for the structural and measurement model: χ^2^/df (238.75/156 = 1.53), GFI (0.91), AGFI (0.88), NFI (0.92), CFI (0.97), and RMSE (0.05). More goodness-of-fit indices for the model are listed in Table 5.

The article "On the networking synthesis of studio factors to the integration of design pedagogy" was retracted in 2025. Reasons: unreliable results or conclusions; concerns about the peer review; concerns about the article.

### 5.2 Testing of the hypothesis

The significance level of the standardised path coefficient was also tested, resulting in levels less than 0.05 or even 0.001 except for the paths from review feedback to design intention and from studio tutorial to design performance (Table 6). As a result (Table 6), the hypotheses about the relationships among the constructs in the final revised model were well supported except H6 and H8; design motivation had a positive effect on design performance; design brief had a positive effect on design motivation; design brief had a positive effect on studio tutorial; design research had a positive effect on design motivation; studio tutorial had a positive effect on design motivation; studio tutorial had no significant effect on design performance; instructor quality had a positive effect on studio tutorial; review feedback had no significant effect on design motivation; review feedback had a positive effect on studio tutorial.

**Table 6:** Hypothesis test and estimates.

Hypothesis		Path coefficient	C.R.	p-value	Result
H1:	DM → GR	0.29***	3.48	<0.001	**Supported**
H2:	DB → DM	0.22*	1.98	0.047	**Supported**
H3:	DB → ST	0.30***	3.55	<0.001	**Supported**
H4:	DR → DM	0.31***	4.52	<0.001	**Supported**
H5:	ST → DM	0.33***	3.10	<0.001	**Supported**
H6:	ST → GR	0.07	0.89	0.372	Rejected
H7:	IQ → ST	0.47***	6.40	<0.001	**Supported**
H8:	RF → DM	0.04	0.32	0.747	Rejected
H9:	RF → ST	0.21*	2.42	0.016	**Supported**

* p < .05

*** p < 0.001

As a result (Fig 2), student performance was affected by design motivation (β = 0.29, standardised path coefficient). Although studio tutorial had no significant influence on student performance (p = 0.37, significant value), it still exerted an indirect positive effect of 0.17 through mediation from design motivation, and 11% of the variance on student performance could be explained in the model (R^2^ = 0.11, coefficient of determination). Through mediation from studio tutorial to design performance, review feedback had an indirect effect of 0.05, and instructor quality had an indirect effect of 0.08 (Table 7). Through mediation effect from design motivation to design performance, design brief had an indirect effect of 0.11, design research had an indirect effect of 0.09, review feedback had an indirect effect of 0.05, and instructor quality had an indirect effect of 0.08 (Table 7).

The article "On the networking synthesis of studio factors to the integration of design pedagogy" was retracted in 2025. Reasons: unreliable results or conclusions; concerns about the peer review; concerns about the article.

**Fig 2:** Path coefficients of the research model after modification by cutting redundant items. (* p < .05; ** p < .05, p < .01; *** p < 0.001).

**Table 7:** Results of the composite path effect.

Construct	Effect	DB	DR	IQ	RF	ST	DM
ST	total	0.30	—	0.47	0.21	—	—
	direct	0.30	—	0.47	0.21	—	—
	indirect	—	—	—	—	—	—
DM	total	0.32	0.31	0.15	0.11	0.33	—
	direct	0.22	0.31	0.00	0.04	0.33	—
	indirect	0.10	—	0.15	0.07	—	—
GR	total	0.11	0.09	0.08	0.05	0.17	0.29
	direct	—	—	—	—	0.07	0.29
	indirect	0.11	0.09	0.08	0.05	0.09	—

Design motivation was jointly affected by design brief (β = 0.22), design research (β = 0.31), and studio tutorial (β = 0.33). Through mediation from studio tutorial, review feedback exerted an indirect positive effect of 0.11, and instructor quality exerted an indirect positive effect of 0.15 (Table 7). In addition, a total of 48% of the variance on design motivation could be explained by those described variables (R^2^ = 0.48).

Studio tutorial was jointly affected by design brief (β = 0.30), review feedback (β = 0.21) and instructor quality (β = 0.47), both explaining 73% of the variance on studio tutorial (R^2^ = 0.73).

## 6. General discussion

There are many issues influencing students' performance in design studio. Contrary to our experience, this research reveals that studio tutorial has no significant effect on student design performance. In design pedagogy, creativity is of critical importance. In recent years, there has been increasing accentuation in the assessment of creativity [52]. As modern society expects higher requirements for education, it is required to change from accumulation of knowledge to the cultivation of creativity. Although final scores are commonly used to identify students' design performance, there is still a debate on this issue. Moreover, the way to improve students' design performance is sometimes uncertain because it involves many external and internal factors. It is more practical to increase students' motivation in professional learning and further trigger their creativity in design practice. Therefore, mobilising students' interest and initiative could enhance the pivot effect that bridges design pedagogy and students' performance in design education.

The article "On the networking synthesis of studio factors to the integration of design pedagogy" was retracted in 2025. Reasons: unreliable results or conclusions; concerns about the peer review; concerns about the article.

Another important finding reveals that the studio tutorial significantly influences students' motivation of participating in their design work. By improving the methodology of design pedagogy, studio tutorial could mediate other factors to stimulate students' participation in their design work. In the proposed model, 48% of the variance on design intention could be explained by the joint influence of design brief (β = 0.22), design research (β = 0.31), and studio tutorial (β = 0.33). If we consider the mediating effect via studio tutorial, the total effect on design motivation from design brief and review feedback is 0.32 and 0.11, respectively (Table 7). Since the evaluation of studio tutorial could be mainly explained (73%) via design brief (β = 0.30), review feedback (β = 0.21) and instructor quality (β = 0.47), the result indicates that the structure of the mainstream studio model is still effective for design education. However, more attention should be paid to establishing a more integrated pedagogy that exerts consistent networking synthesis in all phases to motivate students have more devotion to their design work. The result makes it clear that it’s not possible to isolate a single factor in the process of studio teaching, and training the student to develop a personal capacity to make good, elegant and rational judgements when confronted with a range of complex problems is also very necessary. Purposely forcing students engage in an open dialogue with others about their design decisions is a central tactic of design pedagogy.

For those freshmen just entering college, many are unaware of the essence of professional knowledge and tend to have biased understanding on architecture learning, leading to the dichotomy of regarding architecture either as technical or artistic. Such cognitive fragmentation easily leads to the emergence of learning difficulties. The simplification and idealisation of mental expectations may generate negative impact on their future studies. For junior undergraduates, defining appropriate and acceptable design assignments is necessary. Additionally, it is beneficial to help students gradually tap into creative thinking in a relaxed and enjoyable way, such as observation and mapping via sketching, modelling, recording video, or any other media. Meanwhile, the way of study-in-play and learning-through-making method using the latest technologies such as VR/AR, 3D print and fabrication may ease their anxiety with unfamiliar subjects. Heuristic and guided methods are usually welcome. Casakin [53] finds that novices usually pay more attention to practical aspects, such as fulfilling those given requirements. There should be an awareness of the significant difference between the way novice designers anticipate design products and how experts expect them in a more well-established and cross-disciplinary principle [11]. Therefore, instructors need to communicate with experienced guests who are invited for review to prevent focusing on a junior's innovation and creativity while neglecting their other good potential in design work. Rational design pedagogy is needed both for strengthening communication and eliminating divergences between the perception and evaluation of two parties; it is also needed to help overcome a novice's confusion or passive attitude towards design involvement.

The article "On the networking synthesis of studio factors to the integration of design pedagogy" was retracted in 2025. Reasons: unreliable results or conclusions; concerns about the peer review; concerns about the article.

In the transient sophomore stage, students often show strong interest in adopting new ideas, relying on their experiential understanding and personal preferences to drive the design process and form-making. This open and speculative experimental design stage that calls for trying and testing is an important phase for students to develop abstract thinking via visual aspects. A strong commitment to the original design pushes them to carry out ideas regardless of external circumstances while neglecting external information and references. In this specific situation, the design topic and relevant assignment could be formulated with a detailed plan and timetable. Open questioning and research-oriented topics could allow students to explore the combination of the "found" and "created". They should be encouraged to make their own design research around part of the design task and reprogram the task as necessary. Accordingly, the teaching methods should involve specific research methodologies that encourage students to proceed with design issues at the various stages for complement. Distinct insight and a broad sense of observed phenomena strengthen the conception of design as a cumulative development process, providing a theoretical basis for instructors to integrate research design as a new design methodology for design pedagogy.

Along with the expansion of professional knowledge in the third and fourth years, senior undergraduates evolve deeper understanding towards design philosophy. Their earlier utopian and speculative thinking would encounter more realistic constraints as new information contradict their design ideas, making them adjust how to deal with the conflict between creativity and rationality. If senior students just follow the advice given by the instructor without clarifying for their own understanding and reflection, their design sensibilities would be easily suppressed by self-denial while searching for absolute rationality. Therefore, the ‘pivoting effect’ of studio enhancement should be carefully carried out as all factors work in networking synthesis. At this time, more systematic guidance should be developed with research-oriented programs. When the role of design research is extended, efforts should be made to avoid the so-called ‘wicked problems dilemma’ [54], which leads to deviation from the purpose of the project and time wasting. Students can use design research as a diversion from the process of developing as design solution. Rittel and Webber [54] argued that it’s not possible to develop planning policy simply by engaging in a series of ‘rational’ data-driven design decisions. They advocated an ‘argument-based solution process’, which encourages students to comprehend the complexity of design problem and the social, cultural, and economic aspects behind it. Curiosity and inquisition also promote students' enthusiasm to have autonomous design motivation. Barrett [55] describes a process that "draws on subjective, interdisciplinary and emergent methodologies that have the potential to extend the frontiers of research …a growing recognition of the philosophical and knowledge-producing role of the creative arts in contemporary society needs to be extended both within and beyond the discipline". Insight into the discovery process will spring up as students test and adapt innovative approaches to solve problems, resulting in emergence of more generative concepts. The review process and the feedback to students should include input from scholars and experts in relevant research fields as well as design professionals. They can provide scientific direction in composing ideas, research methods, and the process of argumentation. The latest developments and progress in the related fields could also been introduced, and it is closer to the user-oriented situation in actual design practice. In this way, senior undergraduates formulate a stable pattern of design thinking and expression of their own, which eventually evolves into the foundation for their future work. Such integrated pedagogy relying on studio component networking synthesis could also benefit instructors to gain insights of providing suitable procedural framework and teaching tactics to structure studio management. This could provide a cognitive scaffold to students at all levels of professional development [56].

The article "On the networking synthesis of studio factors to the integration of design pedagogy" was retracted in 2025. Reasons: unreliable results or conclusions; concerns about the peer review; concerns about the article.

## 7. Conclusion

Design work is a complex process involving multivariable problems and various factors which require both clients and designers to reach a consensus. Taking design studio as the subject, this paper uses structural equation modelling and the teaching experience of the authors to interrogate the major factors and their mutual interactions that affect students’ motivation and focus in of architectural design practice. Our findings reveal that studio tutorials and some other exterior factors have insignificant effects on undergraduates' design performance. In contrast, the subjective intention plays an important role in shaping students' behaviours and performance. This finding reveals the importance of transferring exterior forces into internal benefits if the instructor attempts to run the studio in a better way for creative disciplines. The result shows that 48% of students’ intention could be explained by the following factors: design project, research design, review feedback, instructor quality, and studio tutorial. Research oriented design project was validated for its importance as a new trend for design education. Besides, 73% of the effect of studio tutorial could be explained by design brief, review feedback, and instructor quality, indicating the effective structure of the traditional studio. As modern society expects higher requirements for design education, instructors still play a central role; they also must understand what makes undergraduates dedicate to design works. Therefore, creative disciplines and related higher educational institutions should implement strategic efforts to build integrated design pedagogy involving these major factors and networking synthesis by all means.

Although the structural model could stand firm as a whole, only 11% of students’ performance could be explained in this case, indicating a need for further studies with more samples and related factors. Students' performance should be measured not only by the score or even performance only but also by other more valuable aspects. It is a new opportunity to extend our research as the next step, considering both sides of student's and instructor's perspectives, to better understand the complex mechanism of design evaluation. Although beyond the scope of this study, the group comparison among the students in different years could be carried on as an extension in the future.

## Supporting information

S1 Appendix Survey items used in this study. (DOC)

S1 File data_publish. (CSV)
